RETRACTED

# Elevated microRNA-145 inhibits the development of oral squamous cell carcinoma through inactivating ERK/MAPK signaling pathway by down-regulating HOXA1

**DOI:** 10.1042/BSR20182214

**Published:** 2019-06-25

**Authors:** Junhai Ding, Dubin Sun, Pengfeng Xie

**Affiliations:** 1 Department of Stomatology, Affiliated Hospital of Jining Medical University, Jining 272100, P.R. China; 2 Department of Stomatology, Zoucheng People’s Hospital, Zoucheng 273500, P.R. China; 3 Special Functions Section, Jinan Stomatological Hospital, Jinan 250001, P.R. China

**Keywords:** Extracellular-signal-regulated kinase/mitogen activated protein kinase, Homeobox A1, MicroRNA-145, Oral squamous cell carcinoma

## Abstract

**Background:** Oral cancer is one of the most frequent solid cancers worldwide, and oral squamous cell carcinoma (OSCC) constitutes approximately 90% of oral cancers. The discovery of reliable prognostic indicators would be a potential strategy for OSCC treatment. In the present study, we aim to explore the underlying mechanism by which microRNA-145 (miR-145) affected OSCC. **Methods:** Forty-eight patients diagnosed with OSCC were enrolled to obtain the OSCC tissues and adjacent normal tissues. The targeting relationship between miR-145 and Homeobox A1 (HOXA1) was verified*.* In order to assess the effects of miR-145 in OSCC and the detailed regulatory mechanism, the SCC-9 cell line was adopted, in which expression of miR-145 and HOXA1 were altered by transfection. Then, a series of *in vitro* and *in vivo* experiments were performed to evaluate the cell viability, migration, invasion, and tumor growth. **Results:** miR-145 was poorly expressed and HOXA1 was highly expressed in OSCC. HOXA1 was verified as a target of miR-145 to mediate the activation of the extracellular signal-regulated kinase/mitogen activated protein kinase (ERK/MAPK) signaling pathway. In the circumstance of miR-145 elevation or HOXA1 depletion, the SCC-9 cell line manifested with inhibited cell viability, invasion, and migration *in vitro*, coupled with reduced tumor growth *in vivo*, with a decreased expression of ERK/MAPK signaling pathway-related genes/proteins. **Conclusion:** These findings suggested that miR-145 can inhibit HOXA1 to inactivate the ERK/MAPK signaling pathway, thereby suppressing OSCC cell proliferation, migration, and invasion to further inhibit the development of OSCC, highlighting a novel therapeutic target for the OSCC treatment.

## Background

Oral squamous cell carcinoma (OSCC) is one of the most common malignancies all over the world and accounts for over 90% of cancers in the oral cavity [1]. Among all the patients with OSCC, approximately 60% of them suffer from local tumor recurrence and 15–25% of them will develop metastasis [2]. Owing to the lack of understanding of the etiopathogenesis, the survival rate of patients with OSCC in recent 5 years is disappointing, which is less than 50% [3]. OSCC is known as a complex genetic disorder, and previous studies have demonstrated that several dysregulated genes had connection to the growth of OSCC, but the molecular mechanism of OSCC remains to be determined [4,5]. Thereby, new diagnostic and therapeutic approaches to OSCC may be discovered through a better understanding of the molecular mechanisms, which would ultimately contribute to a higher survival rate [6].

RETRACTED

Accumulation of multiple genetic and epigenetic alterations is attributed to the progression of oral carcinogenesis, with an activation of oncogenes and an inhibition of suppressor genes [7]. MicroRNAs (miRNAs), are a class of small non-coding RNAs, that can negatively take control of gene function via binding to complementary sequences in the 3′ untranslated region (UTR) of mRNAs through translational mechanism [8]. Evidence has shown that miRNAs have an impact on the development and progression of OSCC [9]. MicroRNA-145 (miR-145), a major tumor suppressor, which has been proved to express at a low level in diverse epithelial tumors, including lung and breast cancers [10]. In these cancers, miRNAs were found to exert a role through the regulation of Homeobox A1 (HOXA1) [11,12]. HOXA1, an important member of HOXA family, was found to be highly expressed in several malignant tissues and closely associated with tumor progression and poor prognosis [13]. For instance, HOXA1 was a mammary epithelial oncogene in breast cancer and the oncogenic transformation of immortalized human mammary epithelial cells to aggressive *in vivo* carcinoma was caused by adequate expression of HOXA1 [14]. The extracellular signal-regulated kinase/mitogen activated protein kinase (ERK/MAPK) signaling pathway has the ability to regulate multiple biological processes, such as cell growth, apoptosis, proliferation and invasion [15]. Evidence has indicated that miRNAs can exert an anti-angiogenic effect through regulating expression and activity of the MAPK/ERK signaling pathway [16]. Consistently, in our study, in order to find a therapeutic target for the treatment of OSCC, we proposed a hypothesis that miR-145 could hinder OSCC cell invasion and migration and suppress tumor growth through regulation of HOXA1 and the ERK/MAPK signaling pathway.

## Materials and methods

### Study subjects

From August 2012 to December 2016, 48 resected specimens pathologically confirmed as OSCC were collected from Jinan Stomatological Hospital, among which, 21 cases were highly differentiated, 20 cases were moderately differentiated and 7 cases were poorly differentiated or undifferentiated. The patients consisted of 26 males and 22 females with the mean age of 57.5 years (range from 26 to 79 years). There were 15 patients with lymph node metastasis (LNM) and 33 patients without LNM. According to the 2002 TNM classification of International Union Against Cancer (UICC) of oral cancer and oropharyngeal cancer, patients were categorized as 27 cases at stage Ia/Ib and 21 cases at stage IIa/IIb [17]. None of the patients received chemoradiotherapy or other related treatment before the operation. The study was approved by the Institutional Review Board of Jinan Stomatological Hospital (Number 201207003) and written informed consents were obtained from all patients.

RETRACTED

### Cell culture

The tongue squamous cell carcinoma SCC-9 cell lines (CRL-1629, ATCC Manassas, VA, U.S.A.) were cultured in Dulbecco’s modified Eagle’s medium/nutrient mixture F12 (DMEM/F12) (Gibco Island, NY, U.S.A.) containing 10% fetal bovine serum (FBS). When cell confluence reached 80–90% (% refers to g:ml), single cell suspension was obtained by adding trypsin (Gibco Island, NY, U.S.A.). Then cells were centrifuged at 1500 rpm and washed two times with phosphate buffered solution (PBS; pH = 7.4; 0.27 g KH_2_PO_4_; 1.42 g Na_2_HPO_4_; 8 g NaCl, and 0.2 g KCl; 1 l PBS was fully dissolved using 800 ml deionized water and added with concentrated hydrochloric acid until the pH reached 7.4 and the final volume of PBS was 1 l). Cells were then resuspended with the addition of 200 µl PBS. The plate was added with 100 µl anti-human CD44 (Cell Signaling Technology, Danvers, MA, U.S.A., a cell-surface glycoprotein involved in cell–cell interactions, cell adhesion and migration) and cultured for 45 min. After being washed with PBS two times, 200 µl PBS was added to resuspend cells. After CD44 immunofluorescent labeling, cells were categorized using the flow cytometer (FACSCanto II, BD Biosciences San Jose, CA, U.S.A.) and CD44^+^ tumor cells were recollected for cryopreservation or culture for subsequent experiments. Based on experimental data, cells can also be seeded into culture flasks or Petri dishes with different number of wells.

### Cell transfection and grouping

Cells were allocated into the blank group (without any transfection), the miR-145 mimic group (cells transfected with miR-145 mimics; miR-145 mimic refers to the endogenous miRNAs simulating the organism and is chemically synthesized and could enhance the function of the endogenous miRNAs; it is transfected using the same method as the ordinary nucleic acid), the mimic-negative control (NC) group (cells transfected with NC sequence for miR-145 mimics), the miR-145 inhibitor group (cells transfected with miR-145 inhibitors, chemically modified inhibitors to the specific target miRNA), the inhibitor-NC group (cells transfected with NC sequence for miR-145 inhibitors), the siHOXA1 group (cells transfected with siRNA against HOXA1) and the miR-145 inhibitor + siHOXA1 group (cells transfected with combination of miR-145 inhibitors and siRNA against HOXA1; HOXA1 siRNA was transfected using the same method as the transfection of nucleic acid: transfection reagent and HOXA1 siRNA were mixed and added to the culture dishes). Cells were then seeded into a culture bottle (25 cm^2^) and cultured in complete medium (serum-free medium [Thermo Fisher Scientific, California, U.S.A.] supplemented with 10% FBS) until cells reached 30–50% confluence. Five microliters Lipofectamine 2000 (Invitrogen, Carlsbad, CA, U.S.A.) was diluted with 100 µl serum-free medium in an amicrobic Eppendorf (EP) tube. Five minutes later, a total of 1 µg DNA was diluted with 100 µl serum-free medium. Then diluted Lipofectamine 2000 was mixed with diluted DNA. Twenty minutes later, a complex comprising DNA and Liposome was created. Cells in culture bottle were washed with serum-free medium. The complex was added with serum-free medium without the antibiotic and then cells were cultured in the medium at 37°C in an incubator with 5% CO_2_. After 6–8 h, the culture medium was replaced with fresh complete medium for further culture.

RETRACTED

### Reverse-transcription quantitative polymerase chain reaction

SCC-9 cell lines (ATCC® CRL-1629™, human tongue squamous epithelial cells) were transfected for 24 h (Lipo2000 reagent [Thermo Fisher Scientific, California, U.S.A.] was mixed with nucleic acid at 2:1 and put into the culture dishes). After that, the cells were placed on the ice to remove the culture fluid after transfection for 24 h. Total RNA was extracted using TRIzol reagent (Invitrogen, Carlsbad, CA, U.S.A.): cells were washed with D-Hanks solution twice, and 1 ml TRIzol reagent was allowed to stand in the culture bottle for 5 min and transferred to a 1.5 ml EP tube for 5 min; the cells were added with 0.2 ml chloroform and allowed to stand for 5 min, centrifuged at 4°C for 10 min at 12000 rpm; the collected supernatant was transferred to another EP tube, added with 0.5 ml isopropyl alcohol, allowed to stand for 10 min, and centrifuged at 4°C for 10 min at 12000 rpm; with the removal of the supernatant, the cells were added with 1 ml of 70% ethanol, centrifuged at 4°C for 10 min at 7500 rpm, dried for 15 min post the removal of supernatant, and mixed with 20 μl diethylpyrocarbonate (DEPC). Subsequently, RNA was dissolved in ultrapure water with DEPC. The quality of the total RNA was measured in accordance with the absorbance (A) at 260 and 280 nm with ND-1000 spectrophotometer (Nanodrop Technologies, Wilmington, DE, U.S.A.). The RNA concentration was adjusted for reverse-transcription quantitative polymerase chain reaction (RT-qPCR) detection. Then the cDNA was synthesized with reverse transcription kit (Fermentas Inc., Glen Burnie, MD, U.S.A.). TaqMan was used for RT-qPCR detection based on the instruction of the kit (Fermentas Inc., Glen Burnie, MD, U.S.A.). The primer sequences are shown in Table 1. The specificity of the PCR was evaluated using real-time PCR (Bio-Rad, Hercules, CA, U.S.A.). U6 (a kind of stem-loop miRNA exclusively as internal reference) was regarded as the internal reference of miR-145 and β-actin was for the other genes. The mRNA expressions of target gene were calculated by comparing the *C*_t_ value of target gene and *C*_t_ value of reference gene. 2^−ΔΔ*C*_t_^ referred to the relative expressions of target genes and *C*_t_ refers to the number of cycles required to amplify the same products. The experiment was conducted three times.

RETRACTED

**Table 1:** Primer sequences for RT-qPCR

Genes	Primer sequences
*miR-145*	F: 5′-GTCCAGTTTTCCCAGGAATC-3′
	R: 5′-AGAACAGTATTTCCAGGAAT-3′
*U6*	F: 5′-CTCGCTTCGGCAGCACA-3′
	R: 5′-AACGCTTCACGAATTTGCGT-3′
*HOXA1*	F: 5′-ACCCCTCGGACCATAGGATTAC-3′
	R: 5′-AAGGCGCACTGAAGTTCTGTG-3′
*ERK*	F: 5′-GGAAGCATTATCTTGACCAG-3′
	R: 5′-CTCTTGTGTGCGTTGAATGT-3′
*β-actin*	F: 5′-CCAACCGCGAGAAGATGA-3′
	R: 5′-CCAGAGGCGTACAGGGATAG-3′

Abbreviations: F, forward; R, reverse; U6, U6 small nuclear RNA.

### Western blot assay

After transfection for 24 h (transfection reagent was mixed with nucleic acid and added into the culture dish for 24-h culture), the SCC-9 cell lines were collected and added to radio immunoprecipitation assay (RIPA) lysis buffer (Beyotime Biotechnology Co., Ltd., Shanghai, China). The protein concentration was measured using the bicinchoninic acid (BCA) protein assay kit (Thermo Fisher Scientific Inc, Waltham, Massachusetts, U.S.A.), which was stated as follows: BCA working solution was prepared using BCA A solution and BCA B solution at 50:1; after being fully mixed, the BCA working solution was stabilized at room temperature within 24 h; the protein standards were fully dissolved and 10 μl standards were diluted using the same solution as protein samples into 100 μl with the final concentration of 0.5 mg/ml; the protein standards could also be diluted using 0.9% NaCl or PBS; the protein standards (0, 1, 2, 4, 8, 12, 16, and 20 μl) were added to the 96-well plate of protein standards and added with standard diluent until the concentration reached 200 μl; afterward, protein samples were added to the 96-well plate of protein samples and diluted into 20 μl with the addition of standard diluent; each well was added with 200 μl BCA working solution and left undisturbed at 37°C for 30 min or at room temperature for 2 h, or at 60°C for 30 min; the A value would increase as time goes by during the determination of protein concentration and developing reaction would quicken as the temperature goes up; if the protein concentration was relatively low, the proteins could be incubated at relatively high temperatures or the incubation time could be prolonged; the wavelength at A562, 540–595 nm could be measured; the protein concentration was calculated based on the standard curve. Extracted proteins were heated at 100°C for 5 min, and then 20 μg protein was added to each well of a 10% polyacrylamide gel. After electrophoresis at 48 V for 3.5 h, the protein was transferred to a polyvinylidene fluoride (PVDF) membrane. The membrane was blocked with 5% bovine serum albumin (BSA) and placed on a shaking table for 2 h and then washed with Tris-buffered saline with Tween 20 (TBST; pH = 7.4; 0.1% Tween 20) one time. Then 5% BSA (% refers to g:ml) was incubated with the following primary antibodies: HOXA1 (1:1000, ab208781, Abcam), ERK (1:1000, ab52230, Abcam), pERK (1:1000; 3441-100, BioVision), mitogen activated protein kinase (MEK) (1:5000, ab96379, Abcam), pMEK (1:1000, ab96379, Abcam) and GAPDH (1:500, AB181602, Abcam). The dilution ratio refers to the ratio of antibody (μl) to TBS (ml). After washing one time with TBST and putting on the shaking table, the membrane was incubated with secondary antibodies for 1 h, then washed one time with TBST and developed with enhanced chemiluminescence. Images of target protein bands were used for analysis of relative A value. The relative expression of the target protein was expressed as the ratio between A value of the target protein and that of β-actin.

RETRACTED

### Dual-luciferase reporter assay

Online bioinformatics prediction website (microRNA.org) and dual luciferase reporter assays were used to verify the targeting relationship between miR-145 and HOXA1. HOXA1 3′UTR-wild-type (wt) and HOXA1-3′-UTR-mutant (mut) without the binding site of miR-145 were constructed. According to the instructions of TIANamp Genomic DNA kit (Promega Corp., Madison, Wisconsin, U.S.A.), DNA of SCC-9 cell line was extracted. DNA template was used for PCR amplification and purification of HOXA1 and the amplified products of HOXA1-wt and HOXA1-mut were ligated using pGEM-T vector using T4 ligase at 4°C overnight and then transferred to Top10 competent bacteria for screening and identification. Subsequently, HOXA1-wt and HOXA1-mut plasmids were extracted in accordance with the instructions of plasmid extraction kits, followed by double enzyme digestion using endonuclease sites SpeI and Hind III. After purification, the plasmids were connected using T_4_ DNA ligase and luciferase plasmid pMIR-reporter (Huayueyang Biotechnology Co., Ltd., Beijing China) and transformed into DH5α-competent *Escherichia coli*. During extraction, the plasmids were subjected to enzyme digestion and sequencing. The luciferase reporter plasmids with correct sequence (HOXA1-3′-UTR-wt and HOXA1-3′-UTR-mut) were respectively co-treated with miR-145 into SCC-9 cells. After 48 h of treatment, the former culture medium was removed and the cells were washed with PBS twice. Cells in each well were added with 100 μl passive lysis buffer (Promega E1941; ybiotech, Shanghai, China) and violated gently at room temperature for 15 min to collect the cell lysis buffer. The pre-reading time was 2 s, the reading value was 10 s, and the sample size of LARIIStop&Glo® Reagent for each time was 100 μl. The prepared LARIIStop&Glo® Reagent (20 μl/sample) was put into the luminescent tube or plate and measured using bioluminescence detection system (TurnerBioSystems, Sunnyvale, CA, U.S.A.).

### 3-(4,5-dimethyl-2-thiazolyl)-2,5-diphenyl-2-H-tetrazolium bromide assay

When cells reached approximately 80% confluence (% refers to area of cells/total area of the culture dish × 100%), the plate was washed with PBS two times. Cells were treated with 0.25% pancreatin and made into single cell suspension. After calculation, cells were seeded in a 96-well plate with a density of 3–6 × 10^3^ cells in each well (200 μl). Six replicates were prepared and the volume was 200 μl per well. After a period of culture, cells were added with 20 μl MTT (3-(4,5-dimethyl-2-thiazolyl)-2,5-diphenyl-2-H-tetrazolium bromide) (5 mg/ml) (Sigma–Aldrich, St. Louis, MO, U.S.A.) in each well, cultured for 4 h, with the MTT solution aspirated. Then 150 μl of dimethyl sulfoxide (Sigma–Aldrich, St. Louis, MO, U.S.A.) was added into each well and shaken gently for 10 min. A value at 490 nm was measured using an enzyme-linked immunosorbent assay (ELISA) meter at 24, 48 and 72 h. Then a curve showing cell viability was drawn with different time points as abscissa and A values as ordinate.

### Scratch test

A thin wound was created in a six-well plate every 0.5–1 cm. After transfection, 3 × 10^4^ cells were seeded in the six-well plate and cultured overnight. On the following day, when cells grew to approximately 80–90% confluence, vertical wounds were made. After incubation for 48 h, fields with eight wounds were selected randomly from each well, and then images of cell motility were acquired. The relative width was measured using Motic Images Advanced 3.2 software, which can reflect cell migration. Each experiment was conducted three times at least.

RETRACTED

### Transwell assay

The Matrigel (Corning Incorporated, Corning, NY, U.S.A.) was melted at 4°C overnight, diluted (1:3) with serum-free DMEM and then added into each apical chamber (Corning Incorporated, Corning, NY, U.S.A.) in three times (15, 7.5, 7.5 μl) (10 min each time) until all micropores were filled with Matrigel. Cell suspension was seeded into each apical chamber of transwell at a density of 3 × 10^4^ in each well. DMEM (0.5 ml) with FBS was added into basolateral chamber of a 24-well plate. After incubation for 48 h, the number of cells that invaded through the Matrigel matrix was acquired under an inverted microscope. Five fields were selected randomly and the number of invasive cells was expressed with average value. The experiment was conducted three times.

### Xenograft tumor in nude mice

A total of 18 specific pathogen-free (SPF) nude mice aged 4–6 weeks, weighing 16–22 g (Beijing Weitong Lihua Laboratory Animal Technology Co., Ltd, Beijing, China) were housed in SPF laboratory. The conditions were: a laminar air flow room (LAFR) at 22–25°C with a humidity of 55 ± 5%. The food, water and mats were amicrobic. Eighteen nude mice were divided into three groups of six each: blank group, miR-145 mimic group and HOXA1 siRNA group. After disinfection with 75% alcohol, the subcutaneous part of the back of the mice was injected with 0.2 ml SCC-9 cell suspension (10^6^ cells/ml). Following treatment was the injection of the maximum diameter (a) and minimum diameter (b) of the tumors that appeared in mice that were measured every 3 days and the approximate volume of tumor was calculated according to the formula: V = ab^2^/2. The mice were thoroughly observed, whereby special attention was focused on the diet, body shape and defecation of mice. After the injection for 28 days, the mice were killed using cervical dislocation method and grown tumor resected. The size and weight of tumor were measured and then the tumor volume was calculated. The tumor was stored in liquid nitrogen for DNA and protein extraction, which was detected as the above-mentioned procedures. The study protocol was accordance to the Experimental Animal Ethics Committee of Jinan Stomatological Hospital (Number 201706002). All efforts were made to minimize suffering of the animals.

### Statistical analysis

The SPSS 18.0 software (International Business Machines Corporation, Armonk, New York, U.S.A.) was employed for statistical analysis. Normal distribution and equality of variances were tested for all the data. The measurement data which meet the normal distribution were expressed as mean ± standard deviation. The differences between cancer tissues and adjacent normal tissues were compared using paired *t* test and comparisons between two groups were analyzed with independent sample *t* test, which were further adjusted by Welch’s *t* test. Moreover, one-way analysis of variance (ANOVA) was used to compare data among multiple groups, while the pairwise comparison was tested by Tukey. The comparison of data at different time points was analyzed by repeated measurement ANOVA and pairwise comparison was conducted using Dunnett’s test. A *P*-value <0.05 was considered to be statistically significant.

RETRACTED

## Results

### miR-145 expresses at a lower level in OSCC tissues relative to adjacent normal tissues and contributes to OSCC development

We first determined the expression of miR-145 in OSCC and adjacent normal tissues using RT-qPCR and analyzed its relationship with clinicopathological features of OSCC patients to study the function of miR-145 *in vivo*. As shown in Figure 1A, the results showed that the relative expression of miR-145 in OSCC and adjacent normal tissues was 1.094 ± 0.297 and 1.594 ± 0.305, respectively. The results showed that the miR-145 expression was much lower in OSCC tissues than that in adjacent normal tissues (*P*<0.05). In patients with LNM, miR-145 expression was lower than that in patients without LNM (*P*<0.05). Compared with moderately and highly differentiated patients, miR-145 expression in poorly differentiated and undifferentiated patients was decreased significantly. Moreover, miR-145 expression in patients at IIa/IIb stage was found to be down-regulated in comparison with the patients at stage Ia/Ib (all *P*<0.01). However, miR-145 expression showed no correlation with age, gender and tumor location (*P*>0.01) (Figure 1B–F). All the above results implied that miR-145 may be expressed at a low level in OSCC.

**Figure 1:** Poorly expressed miR-145 was found in OSCC tissues relative to adjacent normal tissues (**A**) Relative expression of miR-145 in OSCC tissues and adjacent normal tissues detected by RT-qPCR. (**B**) Relative expression of miR-145 in OSCC patients with different ages detected by RT-qPCR (≥60, *n*=23; >60, *n*=25). (**C**) Relative expression of miR-145 in male and female OSCC patients determined by RT-qPCR (male, *n*=26; female, *n*=22). (**D**) Relative expression of miR-145 in OSCC patients with or without LNM detected by RT-qPCR (patients with LNM, *n*=15; patients without LNM, *n*=33). (**E**) Relative expression of miR-145 in OSCC patients at IIa/IIb and Ia/Ib stages measured using RT-qPCR (patients at Ia/Ib stage, *n*=27; patients at IIa/IIb stage, *n*=21). (**F**) Relative expression of miR-145 in moderately and highly differentiated and poorly differentiated and undifferentiated OSCC patients detected by RT-qPCR (moderately and highly differentiated OSCC patients, *n*=41; poorly differentiated and undifferentiated OSCC patients, *n*=7). The measurement data were expressed as mean ± standard deviation. The differences between OSCC tissues and adjacent normal tissues were analyzed by paired *t* test; *n*=48; comparisons between two groups were analyzed using independent sample *t* test. The experiment was repeated three times.

RETRACTED

### HOXA1 is identified as a target gene of miR-145

Subsequently, we examined whether miR-145 could directly regulate HOXA1 by means of target prediction program and luciferase activity determination. Online bioinformatics prediction software TargetScan implied the target site between HOXA1 and miR-145. Sequences in 3′-UTR binding site between HOXA1 mRNA and miR-145 are shown in Figure 2A. HOXA1-3′-UTR-wt and HOXA1-3′-UTR-mut (specifically directed mutation of the binding site between miR-145 and HOXA1) were constructed to verify that the combination of miR-145 and HOXA1 reduced luciferase activity. SCC-9 cells transfected with miR-145 mimic were divided into two groups: cells co-transfected with wt-miR-145 and HOXA1, and cells co-transfected with mut-miR-145 and HOXA1. Results of the dual luciferase reporter assay demonstrated that in cells carrying the mut-miR-145/HOXA1 plasmid, the luciferase activity did not differ significantly between groups (*P*>0.05). However, luciferase activity reduced to 65% in cells co-transfected with wt-miR-145 and HOXA1 (*P*<0.05) (Figure 2B). The above results indicated that miR-145 might bind to 3′UTR of HOXA1.

**Figure 2:** HOXA1 is a target gene of miR-145 (**A**) Binding site of miR-145 and HOXA1; (**B**) miR-145 binds to the 3′UTR of HOXA1, decreasing the luciferase activity; the measurement data were expressed as mean ± standard deviation; the data between two groups were compared by independent sample *t* test; the experiment was repeated three times; mirSVR refers to thermodynamic stability value (≤ −0.1): lower value suggests stronger binding stability of miRNA–mRNA, and thereby miRNA is more likely to down-regulate the expression of the gene; PhastCons refers to the evolutionary conservation of gene UTR in all species (≥0): the more conservative, the better. *, *P*<0.05 compared with the HOXA1-mut group.

### miR-145 up-regulation or HOXA1 knockdown impairs SCC-9 cell proliferation, migration and invasion

In the following experiments, we mainly investigated the effects of miR-145 and HOXA1 on proliferation, migration and invasion of OSCC cells using MTT assay, Transwell assay and scratch test, respectively.

RETRACTED

The results of MTT assay showed that A values were not significant differences in cell proliferation in the mimic NC (NC of miR-145 mimic), inhibitor NC (NC of miR-145 inhibitor), miR-145 inhibitor + siHOXA1 and blank groups during 24 h (all *P*>0.05) (Figure 3). Cell proliferation in the mimic NC, inhibitor NC, miR-145 inhibitor + siHOXA1 and blank groups showed no difference at 24, 48 and 72 h. After 48 and 72 h, cell proliferation in the miR-145 mimic and siHOXA1 groups was inhibited as compared with the blank group (*P*<0.05). In contrast with the blank group, cell proliferation in the miR-145 inhibitor group was increased (all *P*<0.05).

**Figure 3:** miR-145 overexpression or HOXA1 depletion attenuates OSCC cell proliferation The measurement data were expressed as mean ± standard deviation and analyzed by repeated-measurement ANOVA followed by Dunnett’s post hoc test; the experiment was repeated three times. Abbreviation: siHOXA1, siRNA against HOXA1. * *P*<0.05 compared with the mimic NC group or the inhibitor NC group.

The results of scratch test showed the width (μm) of cell migration: 241.57 ± 24.64 in the blank group, 378.84 ± 38.64 in the miR-145 mimic group, 203.66 ± 21.53 in the siHOXA1 group, 69.53 ± 7.14 in the mimic NC group, 217.05 ± 22.53 in the miR-145 inhibitor group, 392.71 ± 40.52 in the inhibitor NC group, and 265.85 ± 26.67 in the miR-145 inhibitor + siHOXA1 group (Figure 4A,B). Cell migration showed no difference in the mimic NC, inhibitor NC, miR-145 inhibitor + siHOXA1 and blank groups (all *P*>0.05). Compared with the blank group, OSCC cell invasion in the miR-145 mimic group and the siHOXA1 group was inhibited, however, OSCC cell invasion in the miR-145 inhibitor group was promoted significantly (all *P*<0.05).

**Figure 4:** Enforced miR-145 overexpression or reduced HOXA1 inhibits OSCC cell invasion and migration (**A**) Representative images of cell width at 0 and 48 h in each group; (**B**) diagram of width of injury line in each group; (**C**) representative images of cell invasion in each group; (**D**) the number of invasive cells in each group; the measurement data were expressed as mean ± standard deviation and analyzed by one-way ANOVA, followed by Tukey’s post hoc test; the experiment was repeated three times. *, *P*<0.05 compared with the mimic NC group or the inhibitor NC group. Abbreviation: siHOXA1, siRNA against HOXA1.

According to the result of Transwell assay, the number of cells that invaded through the Matrigel matrix into the lower surface of the filter was 39.12 ± 4.11 in the blank group, 22.65 ± 2.54 in the miR-145 mimic group, 46.29 ± 4.76 in the siHOXA1 group, 76.84 ± 8.0 in the mimic NC group, 42.9 ± 5.0 in the miR-145 inhibitor group, 25.19 ± 2.04 in the inhibitor NC group, and 44.95 ± 4.89 in the miR-145 inhibitor + siHOXA1 group (Figure 4C,D). Cell migration showed no difference in the mimic NC, inhibitor NC, miR-145 inhibitor + siHOXA1 and blank groups (all *P*>0.05). Compared with the blank group, cell migration in the miR-145 mimic group and the siHOXA1 group was inhibited, however, cell migration in the miR-145 inhibitor group was promoted (all *P*<0.05).

RETRACTED

Taken together, the above findings suggested that miR-145 up-regulation and HOXA1 knockdown might inhibit SCC-9 cell proliferation, migration and invasion.

### miR-145 up-regulation or HOXA1 knockdown decreases CD44^+^ tumor cells

Furthermore, we sorted the CD44-positive tumor cells using flow cytometry to evaluate the regulatory effects of miR-145 and HOXA1 on OSCC cell invasion and metastasis again. As shown in Figure 5, in contrast with the blank, miR-145 inhibitor + siHOXA1 and mimic NC groups, the proportion of CD44^+^ OSCC cells in the miR-145 mimic group and the siHOXA1 group was decreased (all *P*<0.05). The proportion of CD44^+^ OSCC cells in the miR-145 inhibitor group was significantly increased compared with the blank, miR-145 mimic, mimic NC, inhibitor NC, siHOXA1 and miR-145 inhibitor + siHOXA1 groups (all *P*<0.05). These findings demonstrated that miR-145 might reduce CD44^+^ tumor cells and HOXA1 promote its growth, suggesting that miR-145 can hinder OSCC cell invasion and metastasis.

**Figure 5:** Flow cytometry analysis indicated that miR-145 reduced yet HOXA1 facilitated the growth of CD44^+^ tumor OSCC cells by statistical analysis of ANOVA The measurement data were expressed as mean ± standard deviation and analyzed by one-way ANOVA, followed by Tukey’s post hoc test; the experiment was repeated three times. % refers to the proportion of CD44^+^ cells in total cells. *, *P*<0.05 compared with the mimic NC group or the inhibitor NC group.

### miR-145 negatively modulates HOXA1 and inhibits the activation of ERK/MAPK signaling pathway

The regulatory effects of miR-145 on the ERK/MAPK signaling pathway by mediating HOXA1 were studied by detecting the mRNA and protein expression of the ERK/MAPK signaling pathway-related genes using RT-qPCR and Western blot assay (Figure 6A–C). Based on the results of RT-qPCR and Western blot assay, the results demonstrated that the levels of the ERK/MAPK signaling pathway-related proteins had no significant difference in the mimic NC, inhibitor NC, miR-145 inhibitor + siHOXA1 and blank groups (all *P*>0.05). Compared with the blank and mimic NC groups, the expression of miR-145 was elevated, but the mRNA and protein expression of HOXA1, ERK and MEK as well as the extents of ERK and MEK phosphorylation was significantly decreased in the miR-145 mimic group (*P*<0.05). In contrast with the blank group, the mRNA and protein expression of HOXA1, ERK, and MEK as well as the extents of ERK and MEK phosphorylation were attenuated in the siHOXA1 group (*P*<0.05). Compared with the inhibitor NC group and the blank group, the expression of miR-145 was significantly decreased, while the mRNA and protein expression of HOXA1, ERK, MEK as well as the extents of ERK and MEK phosphorylation was significantly increased in the miR-145 inhibitor group (*P*<0.05). The above results demonstrated that miR-145 might be a negative regulator of HOXA1 and inhibit the activation of the ERK/MAPK signaling pathway.

RETRACTED

**Figure 6:** miR-145 decreased HOXA1 expression and inhibited the activation of the ERK/MAPK signaling pathway *in vitro* (**A**) miR-145 expression and the mRNA expression of HOXA1 in each group; (**B**) protein bands in each group; (**C**) protein levels of HOXA1, ERK, MEK, and the extents of MEK and ERK phosphorylation in each group; the measurement data were expressed as mean ± standard deviation and analyzed by one-way ANOVA, followed by Tukey’s post hoc test; the experiment was repeated three times. *, *P*<0.05 compared with the mimic NC or inhibitor NC group. Abbreviations: p-ERK, phosphorylated-ERK; p-MEK, phosphorylated-MEK; siHOXA1, siRNA against HOXA1.

### miR-145 up-regulation and HOXA1 knockdown suppress tumor growth of OSCC *in vivo*

At last, OSCC SCC-9 xenograft tumors in nude mice were used to detect the effects of miR-145 and HOXA1 on the tumor growth of OSCC *in vivo.* The tumor volume was calculated and the curve of tumor growth was drawn. It was found that as time went by, the tumor volume of mice in the blank group was increased gradually when compared with those of mice in the miR-145 mimic and siHOXA1 groups but the tumor volume of mice in the miR-145 mimic group and the siHOXA1 group had no significant difference (Figure 7A). In the siHOXA1 group, four out of five mice showed induced tumor, while xenograft tumors were formed in the miR-145 mimic and blank groups (Figure 7B). In comparison with the blank group, the tumor size of the miR-145 mimic and siHOXA1 groups was smaller (*P*<0.05), and the miR-145 mimic and siHOXA1 groups showed no significant difference (*P*>0.05). miR-145 expression in miR-145 mimic group was much higher compared with the blank group and the siHOXA1 group (all *P*<0.05) (Figure 7C). Further, it was indicated that the protein expression of HOXA1, ERK, and MEK was down-regulated in the miR-145 mimic group and the siHOXA1 group when in comparison with the blank group (Figure 7D,E). The results showed that miR-145 overexpression or HOXA1 depletion might repress tumor growth of OSCC.

RETRACTED

**Figure 7:** miR-145 up-regulation and HOXA1 knockdown suppressed the growth of xenograft tumors in nude mice (**A**) Changes in tumor volume at 0, 9, 18, and 27 days; (**B**) xenograft tumors in each group; (**C**) relative expression of miR-145 in each group; (**D**) protein bands in each group; (**E**) relative protein levels of HOXA1, ERK, and MEK in each group; the measurement data were expressed as mean ± standard deviation and analyzed by one-way ANOVA; the data among multiple groups at different time points were analyzed using repeated-measurement ANOVA, followed by Dunnett’s post hoc test. Data in different groups were analyzed using one-way ANOVA, followed by Tukey’s post hoc test. *n*=6; the experiment was repeated three times. *, *P*<0.05 compared with the blank group (the nude mice only injected with SCC-9 cell line). Abbreviation: siHOXA1, siRNA against HOXA1.

## Discussion

OSCC is a malignant tumor, which is less sensitive to chemotherapy and is resistant to anticancer drugs because of its high level of hypoxia [18]. In that case, it is desirable to explore new molecular therapeutic targets and discover preventive agents for patients with OSCC through a better clarification of the molecular mechanism and the functional significance [19]. However, considering many potential targets governed by each miRNA, one challenge in understanding functional miRNA contributions in cancer cell behaviors depends on the identification of *bona fide* molecular targets. In the present study, we aim to find out the mechanism by which biological function of miR-145 affects OSCC cells and the effects on HOXA1 gene and the ERK/MAPK signaling pathway.

Initially, we found that miR-145 was reduced in OSCC tissues while HOXA1 was increased in OSCC tissues. Besides, we also found that overexpression of miR-145 or down-regulation of HOXA1 could inhibit OSCC cell proliferation, invasion and migration. Consistent with the observation in our study, Gao et al. [20] demonstrated that miR-145 was poorly expressed in OSCC tissues and cells when in contrast with the non-tumor controls and miR-145 could serve as an underlying diagnostic target for OSCC. miR-145, as a tumor suppressor, has been largely investigated in recent studies, which reveals a wide range of molecular mechanisms of miR-145 in the regulation of cancer cells. For example, Boufraqech et al. [21] provided evidence that miR-145 inhibited cell progression in thyroid cancer. Zhang et al. [22] also revealed that miR-145 decreased cell proliferation in human colon cancer cells and contributed to colon cancer cell apoptosis. Moreover, a study further demonstrated that miR-145 dramatically inhibited cell proliferation and facilities cell apoptosis of OSCC [23]. HOXA1, has been reported to be implicated in tumor progression, and highly expressed HOXA1 was also found in OSCC when compared with healthy oral mucosas [24]. Hence, we suggested that overexpressed miR-145 or down-regulated HOXA1 may inhibit the proliferation, invasion and migration of OSCC cells. In the subsequent experiments, we demonstrated the function of miR-145 on OSCC cells via the ERK/MAPK signaling pathway by targeting HOXA1.

RETRACTED

Based on the target prediction program and the luciferase activity determination, we found that HOXA1 was a putative target gene of and negatively governed by miR-145. HOXA1 was deregulated in small cell lung cancer (SCLC) and the knockdown of HOXA1 using siRNA contributed to decreased chemosensitivity through inducing apoptosis in SCLC cells [25]. Additionally, Pilato et al. [26] found that overexpression of HOXA1 in breast cancer played a vital role in malignant transformation and tumor aggressiveness. In our results, miR-145 up-regulation and HOXA1 knockdown suppress *in vivo* tumor growth of OSCC, which is associated with blocked ERK/MAPK signaling pathway. MAPK signaling pathway is one of the signaling pathways that can be regulated by miR-145 [27]. Wang et al. [28] explained that miR-145 exhibited an antitumor effect in human colon cells via down-regulating the MAPK signaling pathway, with an inhibition of p-ERK expression. Also, Cai et al. [29] showed that miR-145 inhibited cell proliferation by inhibiting IRS1 expression, which resulted in a limitation in the proteins of the MAPK/ERK signaling pathway. Moreover, Bu et al. [30] reported that in OSCC, the ERK/MAPK signaling pathway can make MMP9 activated, thus contributing to the metastasis of OSCC cells. Another study also has illustrated that cell proliferation of OSCC is attenuated via the down-regulation of the ERK signaling pathway [31]. Hence, we suggested that miR-145 may inactivate the MAPK/ERK signaling pathway by targeting HOXA1.

Consistent with the previous studies, we have confirmed that miR-145 is a tumor suppressor and that the overexpression of miR-145 and the knockdown of HOXA1 significantly reduce cell survival, migration, and invasion in OSCC. We have revealed that the tumorigenic activity of miR-145 is mediated by the inhibition of the oncogenic MAPK/ERK signaling pathway through inhibition of HOXA1. These results indicated that miR-145 overexpression and inhibition of the signaling pathway may potentially provide strategic therapeutic applications in OSCC in the future.

RETRACTED

## Abbreviations

ANOVA: analysis of variance
BCA: bicinchoninic acid
BSA: bovine serum albumin
DEPC: diethylpyrocarbonate
EP: Eppendorf
ERK/MAPK: extracellular signal-regulated kinase/mitogen activated protein kinase
FBS: fetal bovine serum
GAPDH: Glyceraldehyde-3-phosphate dehydrogenase
HOXA1: homeobox A1
IRS1: insulin receptor substrate 1
LNM: lymph node metastasis
MEK: mitogen activated protein kinase
miRNA: microRNA
miR-145: microRNA-145
MMP9: Matrix metalloproteinase
MTT: 3-(4,5-dimethyl-2-thiazolyl)-2,5-diphenyl-2-H-tetrazolium bromide
NC: negative control
OSCC: oral squamous cell carcinoma
PBS: phosphate buffered solution
RT-qPCR: reverse-transcription quantitative polymerase chain reaction
SCLC: small cell lung cancer
SPF: specific pathogen-free
TBST: Tris-buffered saline with Tween 20
